This article has been retracted.

# LncRNA SLNCR1 facilitates angiogenesis and tumor growth in melanoma via DNMT1‐mediated epigenetically silencing SPRY2

**DOI:** 10.1111/srt.13910

**Published:** 2024-09-19

**Authors:** Ke Li, Lijun Wu, Jingting Jiang

**Affiliations:** ^1^ Department of Tumor Biological Treatment The Third Affiliated Hospital of Soochow University, Jiangsu Engineering Research Center for Tumor Immunotherapy, Institute of Cell Therapy, Soochow University Changzhou Jiangsu P. R. China; ^2^ Department of Burn and Plastic Surgery The First Affiliated Hospital of Soochow University Suzhou Jiangsu P. R. China; ^3^ Department of Plastic and Aesthetic Surgery The Second Affiliated Hospital of Soochow University Suzhou Jiangsu P. R. China

**Keywords:** angiogenesis, DNMT1, lncRNA SLNCR1, melanoma, SPRY2

## Abstract

**Background:**

The malignancy of melanoma is attributed to its pronounced invasiveness, extensive vascularization, and rapid tumor cell growth and metastasis. LncRNA SLNCR1 is closely associated with a variety of aggressive tumors. However, our understanding of SLNCR1 influences on malignant melanoma growth metastasis mechanism especially proangiogenic mechanism remains unclear.

**Methods:**

The expression of SLNCR1 was evaluated in melanoma tissues, adjacent tissues, melanoma cell lines. The abilities of SLNCR1 on proliferation, migration, and angiogenesis of HUVECs were detected by CCK‐8, flow cytometry, and Western blot assays. The association between SLNCR1, DNMT1, and SPRY2 was assessed by ChIP, RIP, and Western blot assays. The effect of SLNCR1 on tumor growth was determined using a xenograft model in nude mice.

**Results:**

SLNCR1 was confirmed to be highly expressed in melanoma tissues and cells. CM from melanoma cells transfected with sh‐SLNCR1 attenuated proliferation, migration, and angiogenesis of HUVECs. Moreover, loss of SLNCR1 hindered tumor growth and metastasis, as evidenced by reduced tumor size and weight, as well as angiogenesis. Mechanistic studies revealed that SLNCR1 silenced SPRY2 expression, likely through enhancing DNMT1‐mediated DNA methylation of SPRY2 promoter.

**Conclusion:**

SLNCR1 is an oncogene that interacts with DNMT1 to mediate SPRY2 methylation, thereby suppressing SPRY2 expression and promoting the angiogenesis and tumor growth in melanoma. SLNCR1 may serve as a potential target for melanoma treatment.

**Abbreviations**
DNMTs: DNA methyltransferases
lncRNAs: long non‐coding RNAs
MSP: methylation‐specific PCR
RIP: RNA‐binding protein immunoprecipitation
RTK: receptor tyrosine kinase
RT‐qPCR: quantitative real‐time PCR

## 1 INTRODUCTION

Melanoma is a heterogeneous group of malignancies that occur in the skin or mucosa and can develop from congenital or acquired benign nevi.^1^ The pathogenesis of melanoma includes cutaneous photosensitivity, family genetic history, UV exposure, and the immunosuppressive state of the patient. Melanoma is highly malignant with an insidious onset and rapid progression, leading to a 5‐year survival rate of less than 10% and a poor prognosis.^2^, ^3^ Melanoma cells can enhance tumor angiogenesis by inducing the secretion of pro‐angiogenic factors by themselves, or upregulating the expression of pro‐angiogenic ligand receptors secreted on the surface of melanoma cells, triggering the metastatic process.^4^ Therefore, blockade of tumor angiogenesis‐related molecules and signaling pathways has gradually become an antitumor strategy in melanoma.

Aberrant expression of long non‐coding RNAs (lncRNAs) have emerged as an important component in tumorigenesis in multiple cancers, including melanoma. Increasing evidence demonstrated that lncRNAs could regulate the malignant growth and aggressive metastasis of melanoma. Higher expression of lncRNA HOXD‐AS1 was closely correlated with poor prognosis, in addition, inhibition of CASC2 showed a tumor inhibiting effects via EZH2/RUNX3.^5^ In melanoma, lncRNA LENOX enhanced resistance to MAPK inhibition by optimizing mitochondrial function via interacting with RAP2C.^6^ LncRNA CPS1‐IT1 could act as a competing endogenous RNA for BRG1 to reduce Cyr61 expression, thereby hindering EMT and angiogenesis in melanoma cells.^7^ Several studies have reported that tumor cells can accelerate proliferation and invasion to meet their rapid metastatic needs by upregulating lncRNA SLNCR1 expression.^8^, ^9^, ^10^ In addition, lncRNA SLNCR1 has been shown to participate in melanoma Invasion through a conserved SRA1‐like region.^11^ However, the roles of SLNCR1 in tumor angiogenesis, which is critically involved in metastasis, are unknown.

Recently, it has been reported that tumor‐associated lncRNAs are discovered by methods such as genome‐wide lncRNAs profiling, which epigenetically dysregulate downstream genes through differential chromosomal modifications, mainly through genomic DNA methylation.^12^ LncRNAs can act as operons of DNA methylation, thus prompting key signaling pathways during carcinogenesis. DNA methyltransferases (DNMTs) family, especially DNMT1, has been detected to be overexpressed during tumorigenesis in vivo, and studies have suggested that they may have de novo methylated CpG island promoter function, and this function may be one of the mechanisms that inactivate tumor suppressor genes in human cells. DNA methylation analysis of genes associated with multiple cancers revealed a correlation between methylation levels and SPRY2 gene expression, with its promoter exhibiting hypermethylation that favors tumor biological traits.^13^, ^14^, ^15^ A study collected human hepatoma cells Hep3B and Huh7 and revealed that DNMT1 can be recruited to the SPRY2 promoter and first intron to promote SPRY2 promoter methylation, thereby silencing SPRY2expression,^16^ while the mechanism of SPRY2 and DNMT1 proteins in melanoma has not been clearly reported.

Based on the above research background, this study confirmed that SLNCR1 regulated melanoma metastasis and angiogenesis through in vitro and in vivo experiments, and initially explored its possible mechanism of action. The results of this study will provide a new theoretical and experimental basis for the clinical treatment of melanoma.

## 2 MATERIALS AND METHODS

### 2.1 Tissue specimens

Thirty‐five pairs of clinical samples of primary malignant melanoma tumor tissues and adjacent noncancerous tissues were collected. Specimens were obtained from malignant melanoma patients who visited the Third Affiliated Hospital of Soochow University for inpatient surgical resection between 2018 and 2021. All patients voluntarily signed written informed consent for biological research, and none of them had undergone radiotherapy, chemotherapy, and other treatments before operation. All samples obtained in this study were approved by the ethics committee of the Third Affiliated Hospital of Soochow University and abided by the ethical guidelines of the Declaration of Helsinki.

### 2.2 Cell culture and transfection

A total of six types of cells, HEMA, MV3, A375, A875, SK‐MEL‐256, and HUVECs, were used in this study. All cell lines were purchased from Cell Biology of Chinese Academy of Sciences (Shanghai, China) and cultured in 89% DMEM + 10% FBS + 1% Penicillin‐streptomycin culture. The plasmids for sh‐NC, sh‐SLNCR1, vector, and SLNCR1 overexpression were designed and constructed by Beijing synbiotic Gene Technology Co., Ltd. A375 and A875 cells were routinely digested, centrifuged, and seeded into 6‐well plates, and transfected until the cell density reached 60%–70%. All of above sequences were transfected into cells using Lipofectamine 2000 transfection reagent (Invitrogen), and the conditioned medium of each group of cells was collected after shaken and placed in the incubator for incubation for 24 h.

### 2.3 Immunohistochemical staining

After the tissue sections were deparaffinized with xylene and ethanol, they were put into 1% citrate buffer for antigen heat retrieval. After PBS washing, 3% H_2_O_2_ was added dropwise on the tissues, followed by overnight incubation with Ki67 and CD31 antibody. After PBS washing, sections were incubated with secondary antibody on a drop for 20 min and developed with DAB chromogen. Finally, the sections were counterstained with hematoxylin, PBS anti‐blue, neutral resin glue to block the sections, and the pictures were taken under a microscope, and the results of the staining were counted.

### 2.4 Western blot assay

Tissues and cells were collected for protein extraction, centrifuged at 4°C for charging, and protein concentration was measured by BCA method. 10% SDS‐PAGE gels were prepared, loaded at 30 µG protein per well, electrophoresed onto PVDF membranes, blocked in 5% BSA for 2 h. Rabbit primary antibodies against SPRY2, VEGFA, GAPDH (1:2000) were next added and placed on ice at 4°C overnight. The following day, the membrane was washed three times with TBST by first removing the incubation cassette, re‐suspending it at room temperature for 30 min, adding HRP‐conjugated goat‐anti rabbit IgG, and incubating it at room temperature for 2 h. The membrane was washed three times with TBST and developed with chemiluminescent detection after all.

### 2.5 Quantitative real‐time PCR (RT‐qPCR)

Total RNA of tissues and cells was extracted using an RNA kit, and the extracted RNA was reverse transcribed into cDNA following the reverse transcription kit instructions. A qPCR machine was used afterwards to perform the fluorescent quantitative PCR reaction, and the reaction conditions: 95°C for 30 s; 95°C for 5 s, 60°C for 30 s, for a total of 40 cycles. SLNCR1 was calculated using the 2^−ΔΔCt^ method with GAPDH as the internal reference gene. SLNCR1 and SPRY2 primers were designed and synthesized by Shanghai Agilent Bioengineering Co., Ltd. SLNCR1 forward primer: 5′‐ GAG AAC GTG GTG GAA TCA GA‐3′, reverse primer: 5′‐ TCC CAT CCT CTT TCT TGT CC‐3′; SPRY2 forward primer: 5′‐TCG GCA GGT CCC TTT GTC ATC C‐3′, reverse primer: 5′‐TGC AGG TCA ACT GGT GTC GT‐3′; GAPDH forward primer: 5′‐ GGG AAG CTT G TC ATC AAT GG‐3′, reverse primer: 5′‐TGG ACT CCA CGA CGT ACT CA‐3′, respectively.

### 2.6 Subcellular fractionation assay

In order to separate nuclear RNA from cytoplasmic RNA, PARISTM kit (Ambion, AM1921) was employed in line with the protocols of the manufacturer. U6 RNA was utilized as nuclear control and GAPDH as cytoplasmic control. Subcellular fractionation assay was performed in A375 and A875 cells.

### 2.7 Ethynyl deoxyuridine (EdU) incorporation assay

The Cell‐Light EdU Apollo assay kit (Ribobio, Guangzhou, China) was used to detect DNA replication activity. After digestion of the HUVECs, they were seeded in 96‐well plate at a density of 5 × 10^3^/well and the obtained culture supernatants of A375 and a875 cells with different transfection treatments were added. After cells were adherent, EDU working solution (ratio 1000:1) was prepared in DMEM medium, and then 100 µL of it was added in each well and then put into the incubator and incubated for 2 h. After washing with PBS, 100 µL of 4% paraformaldehyde was added to each well to fix the cells, followed by the addition of 100 µL of Apollo staining reaction fluid. After methanol washes, 100 µL of hoechst33342 staining solution was added to each well and subsequently photographed under a fluorescence microscope.

### 2.8 Flow cytometry

HUVECs were collected and counted at 1 per well 1 × 10^6^ cells were seeded in 6‐well plates. The obtained culture supernatants of A375 and A875 cells with different transfection treatments were added to HUVECs after passing through a cell strainer. After 72 h, the 6‐well plates were removed and, after two washes with PBS, cells were trypsinized for 1 min, collected by centrifugation and resuspended to 1 × 10^6^/mL. One milliliter of the cell suspension was taken for centrifugation and fixed overnight using pre‐cooled ethanol at a volume fraction of 70%. After PBS washing again, cells were resuspended in 100 µL RNase a solution in the dark and water bath at 37°C for 30 min. This was followed by the addition of 400 µL PI staining solution and detection using flow cytometry after incubation for 30 min in the dark at 4°C.

### 2.9 ELISA

The concentration of VEGF was measured following the requirements of the VEGF ELISA Kit (R & D system) product insert. A standard curve was plotted after detecting OD values at 450 nm wavelength, and the VEGF concentration in the samples was calculated.

### 2.10 Wound scratch assay

HUVECs were plated within 6‐well plates, and when the cells were fully confluent as a monolayer, the medium was discarded, PBS was washed three times, and the obtained culture supernatants of A375 and A875 cells with different transfection treatments were added to HUVECs after passing through a cell strainer. A scratch was made in the center of cell fusion with a 200 µL of pipette tip. The floating cells were removed by PBS washing three times, and then photographed after the addition of serum‐free medium as a 0 h scratch image. After 48 h, the cells were photographed microscopically.

### 2.11 Tube formation assay

DMEM medium (without FBS) was mixed with Matrigel at a 1:1 ratio and subsequently pipetted into 60 µL of Matrigel dilution in a 96‐well plate and allowed to solidify overnight. HUVEC cells were harvested by digestion and resuspended using HUVECs culture medium without FBS, adjusting the cell concentration to 4 × 10^4^/well. After the conditioned medium of different transfection treatments (100 µL) was mixed with DMEM (50 µL), they were plated on Matrigel and cultured in an incubator. The specimens were taken under a microscope after 4 h, and the number of lumen‐like structures close to closure was counted.

### 2.12 Methylation detection

Bisulfite conversion was performed using the EZ DNA Methylation‐Gold kit (ZYMO Research, Orange, CA, USA) according to the manufacturer's instructions. Bisulfite‐treated DNA was cloned into pGEM‐T (Promega). For each group, 20 clones were sequenced to analyze the SPRY2 promoter.

### 2.13 Chromatin immunoprecipitation (ChIP)

ChIP assay was performed by using the EZ‐ChIP kit (Millipore) according to manufacturer's protocol. Transfected cells were supplemented with 1% formaldehyde and incubated for 10 min to produce DNA‐protein crosslinks. Then, crosslinked chromatin DNA was sonicated to yield chromatin fragments of 200–300 base pairs, and incubated with anti‐DNMT3A, anti‐DNMT3B, anti‐DNMT1 (Millipore) or IgG at 4°C. The precipitated chromatin DNA was amplified by RT‐qPCR assay.

### 2.14 RNA‐binding protein immunoprecipitation (RIP)

EZ‐Magna RIP RNA‐binding protein immunoprecipitation kit (Millipore, USA) was used in RIP experiment. The transfected cells were ruptured by using RNA lysis buffer containing the protease and RNase inhibitors. Cell lysates were added to the RIP buffer containing the magnetic beads coated with antibody complex (Millipore, USA) or lgG overnight. After washing three times, the beads were incubated with proteinase K. TRIzol reagent was used to isolate total RNA from the extracts. The co‐precipitated RNAs were measured by RT‐qPCR analysis.

### 2.15 Methylation specific PCR (MSP)

Bisulfite‐treated DNA was amplified using specific primers for methylated DNA (M‐MSP) and unmethylated DNA (UMSP), respectively by PCR after unmethylated cytosine was converted to uracil to determine the methylation of SPRY2. The amplified DNA fragments were then subjected to 2% agarose gel electrophoresis and images were taken. The primers for Methylated‐MSP and Unmethylated‐MSP are listed below: Methylated‐MSP forward primer: TTT GTA GTG TTT AGT TCG GTT TCG; Methylated‐MSP reverse primer: CAA TAA ATA ACG TCA TAT AAA TCC G; Unmethylated‐MSP forward primer: TTG GTA TTT GGA GAT AAA TTT G; Unmethylated‐MSP reverse primer: CAA TAA ATA ACA TCA TAT AAA TCC A.

### 2.16 Tumorigenesis in vivo

A375 cells were individually transfected with sh‐NC and sh‐SLNCR1 according to experimental requirements and then obtained into the desired cell line. SPF grade male nude BALB/c mice (4–5 weeks old) were randomly selected into sh‐NC and sh‐SLNCR1 groups (*n* = 6) after a week adaptation and were subcutaneously injected with A375 cells transfected with sh‐NC or sh‐SLNCR1, respectively. Cells from each group in logarithmic growth phase were harvested and re‐suspended by adding 2 mL of PBS, and the cells were adjusted to 5 × 10^6^/mL, respectively. Two hundred microliters of cell suspensions were taken individually using a 1 mL syringe and subcutaneously injected 0.5 cm posterior to the right axillary midline in nude mice. Tumor growth changes were evaluated every 5 days. All mice were sacrificed by excessive CO_2_ after 6 weeks of injection, and the tumors were removed and photographed and weighed. Animal experiments were approved and supervised by the Animal Ethics Committee of the Third Affiliated Hospital of Soochow University. All methods were carried out in accordance with relevant guidelines and regulations.

### 2.17 Statistical analysis

Data were analyzed by using statistical product and SPSS 23 software (SPSS Inc., Chicago, IL, USA). Data were presented as mean ± standard deviation. Student's *t*‐test or ANOVA was used to assess the differential expression. A *p* < 0.05 was considered statistically significant.

## 3 RESULTS

### 3.1 High expression of lncRNA SLNCR1 was frequently detected in melanoma

To examine the role of SLNCR1 in melanoma, the expression of SLNCR1 was evaluated in melanoma tissues and adjacent tissues by RT‐qPCR. The expression of SLNCR1 in melanoma tissues was remarkably upregulated compared with adjacent normal tissues (Figure 1A). Additionally, RT‐qPCR was also used to detect the SLNCR1 expression level in melanoma cell lines. As expected, SLNCR1 was highly expressed in MV3, A375, A875, and SK‐MEL‐256 cells compared to HEMA cells (H8) (Figure 1B). A subcellular fractionation assay revealed that SLNCR1 was mainly located in the nucleus (Figure 1C). Further transfection was performed on human A375 and A875 cell lines to construct SLNCR1 overexpression and silencing stable cell lines, and the effect of the constructs on SLNCR1 differentially expressed stable cell lines was verified by RT‐qPCR experiments. RT‐qPCR assay results showed that the introduction of pcDNA‐SLNCR1 or sh‐SLNCR1 induced a significant elevated/reduced of SLNCR1 levels in A375 and A875 cells, respectively (Figure 1D).

**FIGURE 1:** Expression of SLNCR1 was increased in melanoma. (A), (B) RT‐qPCR results analysing SLNCR1 expression in melanoma tissues and cells. (C) Subcellular fractionation assay analysis SLNCR1 in melanoma cell nuclear and cytoplasm distribution. (D) RT‐qPCR and quantification of SLNCR1 in transfected cells. *p < 0.05.

### 3.2 LncRNA SLNCR1 enhanced cell proliferation ability and migration ability of HUVECs

To gain insight into the mechanistic experiments of SLNCR1, conditioned media from A375 and A875 cells with stable downregulation or overexpression of SLNCR1 were collected and then cultured with HUVEC cells. As shown in Figure 2A, the HUVEC proliferation ability of the transfected sh‐SLNCR1 group was obviously lower than that of the sh‐NC group after treatment with A375 and A875 cell conditioned medium, whereas the proliferative activity of cells in SLNCR1 overexpression group was significantly higher than that in control group (Figure 2A). Flow cytometry data displayed that SLNCR1 overexpression caused an increased in the percentage of HUVECs in the phase S, but decreased following SLNCR1silenced (Figure 2B). Further validated by EDU nuclide incorporation assay results, enhanced SLNCR1 contributes to DNA synthesis in HUVECs, vice versa (Figure 2C). Furthermore, the migratory ability of HUVECs was inhibited after treatment with overexpression of SLNCR1 conditioned medium, however, loss of SLNCR1 produced the opposite result (Figure 2D).

**FIGURE 2:** SLNCR1 significantly reduced the proliferation and migratory ability of HUVECs. (A) CCK‐8 assay presented HUVEC proliferation. (B) Flow cytometry detected the cell cycle of HUVECs. (C) EdU assay detected the proliferation ability of HUVEC. (D) Representative images of HUVEC migration and quantification of wound healing ratio. *p < 0.05.

### 3.3 LncRNA SLNCR1 enhanced angiogenic capacity of melanoma cells

To evaluate the effect of SLNCR1 on angiogenesis of melanoma cells, we further utilized HUVECs in vitro for lumen formation assay. After A375 or A875 cell conditioned medium was mixed and cultured with HUVECs, respectively, we found that SLNCR1 overexpression suppressed the cell lumen structure formation ability, while the results in the silencing SLNCR1 group were opposite (Figure 3A). The angiogenesis marker VEGFA was detected by Western blot and ELISA experiments. The results showed a rising trend in VEGFA expression after overexpression of SLNCR1, in contrast to SLNCR1 silencing, which decreased the levels mentioned above (Figure 3B and C).

**FIGURE 3:** SLNCR1 significantly enhanced HUVEC angiogenesis. (A) Representative images of HUVEC proangiogenic ability and quantification of tube formation. (B) ELSIA detected the level of VEGFA. (C) Representative western blot for VEGFA and quantitative determination of VEGFA protein level in HUVECs. *p < 0.05.

### 3.4 SLNCR1 interacted with DNMT1 protein and epigenetically silenced SPRY2

Researchers have universally found that melanoma can be triggered by the canonical Receptor Tyrosine Kinase (RTK) signaling pathway. Sprouty2 (SPRY2) was observed to be a suppressor of RTK signaling pathway, which may play a role in suppressing melanoma development by inhibiting angiogenesis.^17^ We assessed the expression of SPRY2 and figured out SPRY2 expression was notably lower expressed in the melanoma tissues and cells (Figure 4A and B). Importantly, it is well established that dysregulated expression of SPRY2 correlates with their promoter methylation levels. Subsequently, we used online website (http://www.ebi.ac.uk/Tools/seqstats/emboss_cpgplot/) to predict the methylation status of SPRY2, and found out the CpG island methylation status of SPRY2 promoter region (Figure 4C). The traditional view is that DNMT family members have central function on the epigenetic gene regulation and there is a physical interaction between SPRY2 promoter region and DNMT1.^16^ Therefore, we formed a hypothesis that DNMT family members may be involved in the transcriptional inhibition of SPRY2 expression in melanoma. ChIP assay showed that the relative enrichment level of anti‐DNMT1 was remarkably increased in SPRY2 promoter region compared to that in the lgG group (Figure 4D). The results of RT‐qPCR and western blotting showed that the level of SPRY2 was increased by DNMT1 overexpressed and decreased by DNMT1 knockdown (Figure 4E and F).

**FIGURE 4:** SLNCR1 enhanced SPRY2 promoter methylation by binding to DNMT1. (A), (B) RT‐qPCR results analysis SLNCR1 in melanoma tissues and cells. (C) Image of EBI CpGplot website of SPRY2promoter region CpG island analysis. (D) ChIP analysis of the enrichment of DNMT1 on SPRY2 promoter. (E), (F) Representative RT‐qPCR and western blot for SPRY2 and quantitative determination of SPRY2 protein level in A375 cells. (G) RIP analysis of the enrichment of SLNCR1 in DNMT1‐RNA precipitates. (H) Bisulfite sequencing analysis of the effect of SLNCR1 on SPRY2 promoter. (I) MSP analysis of the regulation of SLNCR1 on SPRY2 promoter methylation level. (J) ChIP analysis of the level of DNMT1 enrichment at the SPRY2 promoter by SLNCR1. *p < 0.05.

Accumulating evidence suggested that SLNCR1 suppresses gene transcription through recruiting DNMT1 to the promoter region of target genes. Thus, it is reasonable to postulate that DNMT1 mediates SPRY2 suppression in a SLNCR1‐dependent manner in melanoma. RIP assay showed an enrichment of SLNCR1 in DNMT1‐RNA precipitates (Figure 4G). To explore whether SLNCR1 regulates SPRY2 expression through promoter DNA methylation, we first utilized the bisulfite sequencing to detect CpG methylation and revealed that SLNCR1 knockdown in A375 cells increased the degree of methylation of the SPRY2 promoter (Figure 4H). We performed MSP to further verify the regulation of SLNCR1 on SPRY2 promoter region methylation status and found that the methylation at SPRY2 promoter region was increased following SLNCR1 overexpression, but decreased following SLNCR1 interference (Figure 4I). The analysis of the binding between DNMT1 and SPRY2 by ChIP demonstrated that SLNCR1 interference in A375 cells reduced the recruitment of DNMT1 at SPRY2 promoter region (Figure 4J).

### 3.5 SPRY2 in SLNCR1‐mediated HUVEC cell proliferation, migration, and angiogenesis

To test whether SPRY2 could rescue the inhibitory effect of SLNCR1 silencing on the activities of melanoma cells, SLNCR1 and/or SPRY2 were silenced in A375 and A875 cells and then collect their conditioned medium. Loss of SPRY2 significantly enhanced the capacity of HUVEC proliferation and reduced the percentage of cells in the phase S after incubation with SLNCR1‐silenced A375 and A875 cell conditioned medium (Figure 5A and B). Besides, loss of SLNCR1 impaired DNA synthesis in HUVEC s, which was restored by SPRY2 inhibition (Figure 5C). SPRY2 interference also abolished the inhibitory effect of SLNCR1 silenced on cell migration (Figure 5D). In addition, the cell lumen structure formation ability by SLNCR1 inhibition was abrogated by SPRY2 silenced (Figure 5E). Likewise, SPRY2 silenced reversed the effect of SLNCR1interference on VEGFA levels (Figure 5F and G).

**FIGURE 5:** SPRY2 involved in SLNCR1‐mediated HUVEC cell proliferation, migration, and angiogenesis. (A) CCK‐8 assay presented HUVEC proliferation. (B) Flow cytometry detected the cell cycle of HUVECs. (C) EdU assay detected the proliferation ability of HUVEC. (D) Representative images of HUVEC migration and quantification of wound healing ratio. (E) Representative images of HUVEC proangiogenic ability and quantification of tube formation. (F) ELSIA detected the level of VEGFA. (G) Representative western blot for VEGFA and quantitative determination of VEGFA protein level in HUVECs. *p < 0.05.

### 3.6 Loss of SLNCR1 prevented the growth of melanoma

To investigate the therapeutic effects of SLNCR1 inhibition on melanoma, a mouse melanoma model was established using A375 cells transfected with sh‐SLNCR1 or sh‐NC. Inhibition of SLNCR1 remarkably restrained the size and weight of tumors at the end of experiments (Figure 6A–C). Tumor growth is dependent on angiogenesis, so we speculated that SLNCR1 might regulate melanoma growth by affecting angiogenesis‐related genes in tumor tissues. After interference of SLNCR1, the expression of SLNCR1, SPRY2, and VEGFA protein was decreased in the sh‐SLNCR1 group (Figure 6D and E). The levels of Ki67 and CD31 levels in sh‐SLNCR1 group were lower than those in sh‐NC group (Figure 6F). Moreover, inhibition of SLNCR1 attenuated MVD values (Figure 6G).

**FIGURE 6:** SLNCR1 inhibition prevented the growth of melanoma. (A) Representative photomicrographs of tumors. (B), (C) Quantitative analysis of tumor size and weight. (D) RT‐qPCR and quantification of SLNCR1 in tumors. (E) Representative western blot for SPRY2 and VEGFA and quantitative determination of SPRY2 and VEGFA protein level in tumors. (F) Representative images of IHC of Ki67 and CD31 in tumors. (G) Quantification of MVD values in tumors. *p < 0.05.

## 4 DISCUSSION

Malignant melanoma is highly lethal with early metastasis. Traditional surgical treatments do not prolong survival time, and response rates to targeted and immunotherapy are low. Studies have shown that targeted and immunotherapy can improve the survival rate of patients, but the response rate of patients to it is not high in clinic, which limits its therapeutic effect to some extent.^18^ Therefore, exploring better treatment strategies is still one of the difficult problems at this stage. Scientists have proposed that the growth and survival of solid tumors are dependent on angiogenesis.^19^ When a tumor grows to 1–2 mm in diameter, it needs to form neovessels to supply itself with nutrients and clear metabolites. Blood vessels in tumors are different from normal vessels both structurally and functionally, and the increased tube wall permeability provides a structural basis for distant metastasis of tumor cells. Therefore, unlike traditional therapies, blocking tumor angiogenesis is also an approach for treating tumors.

LncRNA SLNCR1, also known as linc00673, is a newly identified lncRNA. In vivo and in vitro evidence showed that SLNCR1 was closely related to breast cancer, and YY1 directly bound to the promoter region of SLNCR1 and enhanced the expression level of SLNCR1, leading to the proliferation of breast cancer cells and tumor growth.^8^ Loss of the p53 tumor suppressor gene in lung adenocarcinoma contributed to cell cycle arrest and senescence mediated by SLNCR1 overexpression.^20^ Research scholars collected 71 cases of colorectal cancer tissues, SLNCR1 was detected to be highly expressed in 51 of these tissues, and was positively correlated with tumor malignant metastasis and poor prognosis of patients.^21^ Interestingly, in melanoma, SLNCR1 mediated malignant melanoma invasion and proliferation in an androgen independent manner or transcriptionally activates MMP9, thereby potentially contributing to the high incidence of malignant melanoma metastasis and poor survival in men.^11^, ^22^ Tumor growth and metastasis are known to be dependent on angiogenesis, however, how SLNCR1 affects melanoma metastasis and angiogenesis is poorly understood. The biological behavior of HUVECs was uncovered to be affect tumor cell metastasis and angiogenesis. In this study, we used the supernatant of SLNCR1 differentially expressed cells to culture HUVECs, and the results further confirmed that SLNCR1 can regulate melanoma angiogenesis by promoting the proliferation and migration of HUVECs. Further, in this study, microtubule formation, ELISA and other experiments were performed, and overexpression of SLNCR1 promoted microtubule formation and upregulated the expression level of VEGF, all suggesting that SLNCR1 could promote neovascularization ability.

SPRY2, belonging to SPRY family members, is a regulator of RTK signaling pathways and has recently been implicated as a tumor suppressor in a variety of cancers. Sanchez et al. and Frank et al. found that in diffuse large B‐cell lymphoma SPRY2 promoter hypermethylation, correlated with a significant reduction in 5‐year survival, and expression of SPRY2 could inhibit B‐cell proliferation.^23^, ^24^ In multiple myeloma cells, overexpression of SPRY2 decreased vascular endothelial growth factor secretion, increased ERK inhibitor sensitivity in vitro, and inhibited tumor formation in vivo.^25^ Low gene expression of SPRY2 in breast cancer tissues correlated with increased pathological grade as well as high expression of HER2; In trastuzumab treated patients, low SPRY2 expression was associated with an increased risk of death.^26^, ^27^ Liu et al. revealed that SPRY2 has a more effective inhibitory effect on melanoma than SPRY1, which can inhibit ERK1/2 phosphorylation mediated cell proliferation and melanoma growth.^28^ Importantly, SPRY2 was observed to be a suppressor of RTK signaling pathway, which may play a role in suppressing melanoma development by inhibiting angiogenesis.^17^ Here, we have found through various experiments that SLNCR1 can recruit DNMT1 to the promoter region of SPRT1, which is consistent with previous literature reports. A recent study showed that SLNCR1 reduced p53 expression in papillary thyroid cancer by interacting with DNMT1.^29^ Other studies have shown that SLNCR1silencing inhibits proliferation and drug resistance of prostate cancer cells via decreasing KLF4 promoter methylation.^30^ Therefore, we hypothesized that the molecular mechanism of SLNCR1's role in the angiogenesis of melanoma might be related to SPRY2. To confirm this hypothesis, we silenced SPRY2 after knocking out SLNCR1 in melanoma cells, and found that the silencing of SPRY2 reversed SLNCR1 mediated proliferation, migration, and angiogenesis as well as tumor growth.

In conclusion, we preliminarily confirmed that the promotion of SLNCR1 on the growth and angiogenesis of experimental melanoma is achieved through the DNMT1/SPRY2 pathway. Our research provides a theoretical basis for further regulation of the mechanism of SLNCR1 in melanoma, and provides an experimental basis for the treatment of melanoma.

## CONFLICT OF INTEREST STATEMENT

No conflicts of interest exits in the submission of this manuscript.

## Data Availability

All the data obtained in the current study were available from the corresponding authors on reasonable request.
